# p63 and p73 Transcriptionally Regulate Genes Involved in DNA Repair

**DOI:** 10.1371/journal.pgen.1000680

**Published:** 2009-10-09

**Authors:** Yu-Li Lin, Shomit Sengupta, Katherine Gurdziel, George W. Bell, Tyler Jacks, Elsa R. Flores

**Affiliations:** 1 Department of Molecular and Cellular Oncology, Graduate School of Biomedical Sciences, The University of Texas M. D. Anderson Cancer Center, Houston, Texas, United States of America; 2 Department of Biology and Koch Institute for Integrative Cancer Research, Massachusetts Institute of Technology, Cambridge, Massachusetts, United States of America; 3 Whitehead Institute for Biomedical Research, Cambridge, Massachusetts, United States of America; 4 Howard Hughes Medical Institute, Chevy Chase, Maryland, United States of America; Stanford University School of Medicine, United States of America

## Abstract

The *p53* family activates many of the same genes in response to DNA damage. Because *p63* and *p73* have structural differences from *p53* and play distinct biological functions in development and metastasis, it is likely that they activate a unique transcriptional network. Therefore, we performed a genome-wide analysis using cells lacking the *p53* family members after treatment with DNA damage. We identified over 100 genes involved in multiple pathways that were uniquely regulated by p63 or p73, and not p53. Further validation indicated that *BRCA2*, *Rad51*, and *mre11* are direct transcriptional targets of p63 and p73. Additionally, cells deficient for *p63* and *p73* are impaired in DNA repair and *p63+/−;p73+/−* mice develop mammary tumors suggesting a novel mechanism whereby p63 and p73 suppress tumorigenesis.

## Author Summary

*p63* and *p73* have been identified as important suppressors of tumorigenesis and metastasis. Although they are structurally similar to *p53*, they have many functions that are unique including roles in development and metastasis. Here we show, using a genome-wide analysis of cells lacking *p63* and *p73* individually and in combination, that p63 and p73 regulate many unique target genes involved in multiple cellular processes. Interestingly, one of these pathways is DNA repair. Further validation of differentially expressed target genes in this pathway, revealed that p63 and p73 transcriptionally regulate *BRCA2*, *Rad51*, and *mre11* providing a novel mechanism for the action of p63 and p73 in tumor suppression. These findings have important therapeutic implications for cancer patients with alterations in the p63/p73 pathway.

## Introduction

*p53* acts as a tumor suppressor gene by transcriptionally regulating a multitude of target genes in response to DNA damage [1]. Induction of these genes results in multiple cellular fates including apoptosis and cell cycle arrest. *p63* and *p73* share some of the same functions as *p53*; however, *p63* and *p73* are structurally more complex containing multiple isoforms [2],[3],[4]. The TA isoforms are structurally more like *p53* and contain a transactivation domain while the ΔN isoforms lack this domain and are transcribed from an internal promoter unique to these isoforms [3],[5]. Based on the fact that the TA isoforms are more similar structurally to *p53*, the TA isoforms were hypothesized and shown to be the major isoforms that induce transcription and are thought to have tumor suppressive functions [3],[5],[6],[7],[8]. In contrast, the ΔN isoforms have been shown to act as dominant negatives against the TA isoforms of *p63* and *p73* and also against *p53*. Because of the ability of the ΔN isoforms to act as dominant negatives and their overexpression patterns in human tumors [2],[6],[9],[10],[11], these isoforms have been hypothesized to act as oncogenes [3],[5],[6]. Interestingly, recent data have revealed that the ΔN isoforms of *p73* can induce apoptosis, cell cycle arrest and transactivate target genes, such as *p21, 14-3-3σ*, and *GADD45* [12]. Additional studies have demonstrated that expression of ΔNp73β at physiological levels can result in the suppression of cell growth in the presence or absence of *p53* indicating that this isoform of *p73* may act as a tumor suppressor gene [12]. Similarly, the ΔN isoforms of *p63* have also been shown to have the ability to transactivate target genes [13]. In the case of *p63*, the ΔN isoforms are more highly expressed in epithelial tissues [14], and thus it is not be surprising that the ΔN isoforms transcriptionally regulate genes involved in the morphogenesis and differentiation of the epithelium. Given the structural complexity and expression of p63, p73, and their isoforms, the transcriptional targets of these genes are an area of growing research.

We and others have shown previously that *p63* and *p73* can induce apoptosis in response to DNA damage [2],[8],[15]. Many of the target genes induced by *p63* and *p73* are shared with *p53* [2],[8]. Additionally, we have shown that the *p53* family of genes is interdependent on each other in the apoptotic response and in the suppression of tumorigenesis. *p53+/−;p63+/−* and *p53+/−;p73+/−* develop some of the same tumor types as *p53+/−* mice, but the phenotype of the tumors in the compound mutant mice is highly aggressive and metastatic indicative of cooperativity between family members [7],[15]. Mice heterozygous for combinations of the *p53* family members develop a novel tumor spectrum compared to *p53+/−* mice indicative of functions of *p63* and *p73* independent of *p53* [7]. These independent functions suggest that p63 and p73 may have unique transcriptional programs.

To understand the transcriptional program of p63 and p73, we made use of MEFs deficient for each of the *p53* family members individually and in combination and performed a genome wide analysis using cDNA microarray analysis to determine whether p63 and p73 transcriptionally regulate genes independently of p53 in response to DNA damage. Interestingly, we found that p63 and/or p73 transactivate sets of genes independent of p53. Among these sets of genes are those involved in homologous DNA repair, including *Rad51*, *BRCA2*, *mre11* and *Rad50*. p63 and p73 were found to bind to these gene promoters by ChIP assay and to transactivate them as demonstrated by luciferase assay. Surprisingly, the ΔN isoforms of *p63* and *p73*, which have been shown to be weak transactivators, transactivate the *Rad51* and *BRCA2* genes to high levels. In addition, *p63−/−, p73−/−* and *p63−/−;p73−/−* MEFs exhibited an impaired ability to repair their DNA and to survive in a clonogenic survival assay. Additionally, *in vivo* evidence from *p63/p73* mutant mice supports this finding; *p63+/−;p73+/−* mice develop mammary adenocarcinomas at a high frequency [7]. Here, we show that these mammary tumors lose expression of p63, p73, BRCA2, and Rad51. Our findings indicate that p63 and p73 may suppress tumorigenesis by transcriptionally regulating critical genes in the DNA repair pathway.

## Results

### The *p53* family of genes cooperates and acts independently in the regulation of transcriptional targets

The *p53* family members, *p63* and *p73*, have previously been shown to share many of the same target genes as *p53* [2],[8]. Additionally, both p63 and p73 have the ability to bind to the p53 consensus binding site. *p63* and *p73* also have biological activities independent of *p53*. Consequently, we were interested in determining whether *p63* and *p73* had unique transcriptional target genes. A cDNA microarray analysis was performed using E1A expressing MEFs deficient for each *p53* family member individually (*p53−/−, p63−/−, p73−/−*) and in combination (*p63−/−;p73−/−*). These cells were treated with doxorubicin, a DNA damaging agent, to induce apoptosis in wild-type E1A MEFs. *p53−/−* and *p63−/−;p73−/−* E1A MEFs have previously been shown to be resistant to this treatment while the *p63−/−* and *p73−/−* E1A MEFS are partially resistant to apoptosis [15]. Microarray analysis revealed a large number of genes differentially expressed in the MEFs deficient for each *p53* family member. Because we were interested in identifying genes that are transactivated by the *p53* family members in response to DNA damage, genes that are down regulated in the absence of the *p53* family members were further analyzed.

After filtering and statistical analysis using SAM [16], 620 out of 15,488 genes were found to be down regulated in at least one of the single knockout E1A MEF lines compared to wild-type E1A MEFs in response to DNA damage. Eight-six of the 620 genes were down regulated in the *p53−/−*, *p63−/−*, and *p73−/−* E1A MEFs as illustrated by the Venn diagram (Figure 1 and Figure S1). There were also sets of genes that were uniquely regulated by each *p53* family member; the *p53−/−*, *p63−/−*, and *p73−/−* MEFs each had 109, 148, and 131 genes down regulated respectively. Lastly, there were sets of genes that were regulated by two family members only; forty-seven were down regulated in the absence of *p53* and *p63*, 41 in the absence of *p53* and *p73*, and 58 in the absence of *p63* and *p73*. The final list of differentially regulated genes was processed through multiple bioinformatic pipelines to identify biological pathways regulated by the *p53* family members. Pathway analysis using the web-based KEGG, BioCarta, and GenMAPP databases indicated that the p53 family members regulate numerous pathways including: cell cycle, DNA-damage, p53 signaling, apoptosis, ribosomal proteins, metabolic pathways, and growth factor signaling (Table S1).

**Figure 1:** Venn diagram illustrating genes down regulated in the absence of the *p53* family members. Eighty-six genes (brown) were down regulated in the absence of all three *p53* family members. A number of genes were down regulated in the absence of each *p53* family member individually; 109 in *p53* deficient cells (red), 148 in *p63* deficient cells (yellow), and 131 in *p73* deficient cells (blue). Several genes were down regulated in the absence of two family members; 47 in the absence of *p53* and *p63* (orange), 58 in the absence of *p63* and *p73* (green), and 41 in the absence of *p53* and *p73* (purple).

The putative target genes identified by microarray analysis were analyzed for the presence of a p53 or p63 consensus binding sites using a computer based genome wide search and HMMER1 software [17]. The promoter sequences (defined as 5 kb upstream and downstream of the transcription start site excluding exons) from the 724 down regulated genes were queried, and 700 of these genes were found to have p53 family member motifs. Of these, 669 genes contained p53 family member motif sites with the ideal p53 spacer of 6 nucleotides between the two half sites. Scores were then given to each identified binding site corresponding to how well they matched with previously published p53 or p63 matrices (Table S2).

Hierarchical clustering was then performed in the specified knock out MEFs relative to wild-type after DNA damage to highlight patterns between the downregulated genes in the *p53−/−*, *p63−/−* and *p73−/−* E1A MEFs (Figure 2 and Figure S1). Interestingly, many genes were differentially regulated in the various MEF lines (Figure 2) indicating that p63 and p73 have unique target genes. Also, many genes were found to be down-regulated in all mutant cell types supporting the hypothesis that all three transcription factors can transactivate some of the same gene targets (Figure 2).

**Figure 2:** Heatmap showing unsupervised hierarchical clustering analysis of *p53*, *p63*, and *p73−/−* E1A MEFs after doxorubicin treatment. Each row represents the specified gene. Each column represents the expression level of a specified knock out MEF line relative to the expression level of wild-type MEFs after DNA damage. The red color indicates upregulation, the green color indicates down regulation, while black indicates no significant change of the indicated gene expression. Clustering based on Euclidean distance indicates that *p63-* and *p73-*deficient E1A MEFs are more similar to each other than to *p53−/−* E1A MEFs. Genes of interest are listed in boxes and are associated with their corresponding location on the heatmap.

DNA damage triggers numerous cellular responses including an extensive DNA repair pathway involving numerous genes [18]. Microarray analysis revealed that the *p53* family members regulate numerous genes involved in the DNA repair pathway. Many of these genes seemed to be uniquely regulated by *p63* and/or *p73*. After DNA damage, loss of *p63* or *p73* prevents induction of *Brca2* (Figure 2, cluster 4), an essential co-factor in Rad51-dependent DNA repair of double-stranded breaks, and *Rad51* itself (Figure 2, cluster 3) [18]. Sequence analysis also indicates that p53/p63 response elements exist in both the promoter and intronic region of *Brca2* and *Rad51* (Table 1 and Table S2). Clustered with *Rad51* are *Dbf4*, a regulator of *Cdc7* and a prognostic determinant for melanoma development, and *Gas6*, which cooperates with the tyrosine receptor kinase *Axl* in tumor proliferation and cell survival (Figure 2, cluster 3). We also found additional genes that were uniquely down-regulated in *p63−/−*, *p73−/−*, and *p63−/−;p73−/−* MEFs. These hits indicate that *p63* and *p73* have roles independent of *p53* in the DNA-damage response pathway. For example, expression of *Rad50*, which forms a complex with mre11 and Nebrin, is found to be down regulated in *p63−/−;p73−/−* MEFs relative to wild-type MEFs treated with doxorubicin. There are also p53 family response elements upstream of the transcription start site of *Rad50* (Table S2).

**Table 1:** *p53* family response elements assayed by ChIP.

Element	Intron	Sequence	MM/spacer	Binding
RAD51-1	1 : −1766	a**t**gCTTGcc**a** a**c**aCTTG**a**tt	4/0	none
RAD51-2	1 : −220	**ctc**CTAG**aa**c tgaagttataa a**c**aCATG**aa**t	8/11	p73
RAD51-3	2 : +867	aaaCAAGcc**a** c aaaCAAGt**ag**	3/1	p73
RAD51-4	2 : +1347	gagCTTG**g**t**g** g**c**aCTTGctt	3/0	none
BRCA2	2 : +133	ag**t**CAAG**g**t**g** a a**t**gCTTGctt	4/1	p63 & p73
MRE11-1	1 : −744	**t**ggCTTGt**gg** cctccctggtcgactc **t**gaCAAGtcc	4/16	none
MRE11-2	1 : −712	g**tc**CATGtt**g** ggtaacttaggctttgctac gg**t**CTTGt**ag**	6/20	none
MRE11-3	1 : −171	g**c**gCTTGttc aaaaagtctaccctgcaactga g**ct**CATGtt**a**	4/22	p63

Shown are the sequence elements assayed by ChIP analysis. Mismatches are shown in bold-face type.

The intron number and location are shown for each element. MM denotes the number of mismatches to the p53/p63 consensus binding site, spacer indicates the number of nucleotides within the spacer region of the putative binding site, and the binding column shows which family member bound to the element by ChIP assay.

In addition to genes that are uniquely regulated by *p63* and/or *p73*, genes controlled by all three *p53* family members were identified. *Mre11*, a gene that functions in the repair of DNA double strand breaks, was found to be down-regulated in *p53*, *p63*, and *p73* deficient E1A expressing MEFs (Figure 2, cluster 1). In addition, sequence analysis revealed multiple p53/p63 response elements (Table S2). Genes with similar expression profiles as *mre11* include the growth factor signaling components *Ghr* and *Sos1* as well as the apoptotic components *Traf1* and *Cathepsin D* all of which contain p53 family member binding sites (Figure 2, cluster 1 & 6 & Table S2).

Multiple genes involved in other biological processes, including tumor progression, metastasis and development were found to be differentially regulated in the various E1A MEF cells. For example, *Mmp2*, a gene shown to play a role in embryonic development and tumor metastasis, is also down regulated in the absence of *p73* after doxorubicin treatment. Clustered with *Mmp2* are many signaling components such as *Grb2*, *Stat1*, *Map3k14*, and *Mapk8ip3*- all of which have at least one *p53* family member binding motif present near its promoter (Figure 2, cluster 5 and Table S2). Interestingly, *brachyury*, the developmental transcription factor, was identified as a putative *p63* target gene (Figure 2, cluster 2). Given the identified roles of brachyury in limb development, cancer, and hematopoetic stem cells and the development phenotype of the *p63−/−* mouse, this putative target has important biological significance [19],[20],[21],[22]. We found *brachyury* to contain multiple p53 family response elements both upstream of its transcriptional start site and within the first intron (Table S2). Other *p63* dependent genes that cluster with *brachyury* include *Abr*, the GAP for the small GTPase Rac, *Socs3*, involved in cytokine and apoptotic signaling, and the zinc-finger transcription factor *Klf9* which is implicated in control of cell proliferation, cell differentiation, and cell fate (Figure 2, cluster 2).

### Genes involved in DNA repair are not induced in response to DNA damage in the absence of *p63* and/or *p73*

Strikingly, the results from the cDNA microarray indicate that genes in the DNA repair pathway are differentially regulated in MEFs lacking *p63* and/or *p73* after treatment with DNA damaging agents. To verify these putative transcriptional targets of p63 and p73, quantitative real time PCR was performed. The expression of *mre11*, *BRCA2*, *Rad51*, and *Rad50* was examined in wild-type, *p53−/−*, *p63−/−*, *p73−/−* and *p63−/−;p73−/−* E1A MEFs before and after treatment with doxorubicin for 12 hours and 5 Gy of gamma radiation. Interestingly, *mre11*, *BRCA2*, *Rad51*, and *Rad50* are all induced in wild-type E1A MEFs after these treatments (Figure 3). We measured the baseline levels of mRNA of *mre11*, *BRCA2*, *Rad51*, and *Rad50* to determine levels of these transcripts prior to DNA damage (Figure S2). After treatment with doxorubicin or gamma radiation, levels of *mre11* mRNA are not induced to wild-type levels in *p63−/−*and *p63−/−;p73−/−* E1A indicating that p63 may transcriptionally regulate this gene (Figure 3). Similarly, the levels of BRCA2 are significantly lower in *p73−/−* and *p63−/−;p73−/−* E1A MEFs than in wild-type or *p53−/−* E1A MEFs (Figure 3) after treatment with doxorubicin and gamma radiation. Likewise, the *Rad51* gene is not induced to wild-type levels in *p63−/−*, *p73−/−*, and *p63−/−;p73−/−* E1A MEFs after treatment with DNA damaging agents (Figure 3), indicating again that *p63* and *p73* may be critical transcriptional activators of Rad51 after DNA damage. Lastly, Rad50 also showed a pattern indicative of transcriptional regulation by both *p63* and *p73*. The mRNA levels of Rad50 are approximately 4-fold lower in *p63−/−;p73−/−* E1A MEFs than in wild-type E1A MEFs (Figure 3) after treatment with doxorubicin and gamma radiation. Taken together, these data indicate that *mre11*, *BRCA2*, *Rad51*, and *Rad50* may be transcriptional targets of *p63* and *p73* in response to DNA damage.

**Figure 3:** Genes involved in DNA repair are differentially expressed in MEFs deficient for *p63* and/or *p73*. Real time PCR analysis of E1A MEFs of the following genotypes (wild-type, *p53−/−*, *p63−/−, p73−/−* and *p63−/−;p73−/−*) after treatment with (A) doxorubicin (0.34 µM) for 12 hours or (B) γ radiation (12 hours). The Y-axis shows the fold induction. Bars represent 3 MEF lines for each genotype, each performed in triplicate. Data represent the mean ± SEM. The asterisk denotes statistical significance compared to wild-type, p<0.001.

### Loss of *p63* and *p73* in mice results in mammary adenocarcinomas with low expression of BRCA2 and Rad51

As previously reported, twenty percent of mice heterozygous for *p63* and *p73 (p63+/−;p73+/−)* develop mammary adenocarcinomas [7] (Figure 4), and ninety percent of these tumors lose the wild-type allele of *p63* and *p73* [7]. Given that *BRCA2* plays an important role in the pathogenesis of mammary adenocarcinoma, this made it a relevant biological target for p63 and p73 in mammary tumors. The protein levels of Rad51 was first examined by Western blot analysis using wild-type and *p63−/−;p73−/−* MEFs. Interestingly, the basal level of Rad51 is lower in *p63−/−;p73−/−* MEFs compared to wild-type MEFs (Figure 4A). The levels of Rad51 in *p63−/−;p73−/−* MEFs are not induced in response to gamma irradiation; however, a 2-fold increase in expression of Rad51 was detected in the wild-type MEFs after DNA damage. To determine whether this change in expression pattern of Rad51 was cell-type specific, we performed immunohistochemistry on mammary adenocarcinomas from *p63+/−;p73+/−* mice where LOH of *p63* and *p73* had occurred (n = 10) (Figure 4F–4I). Indeed, Rad51 as well as BRCA expression is detected in normal mammary glands (n = 10) of *p63+/−;p73+/−* mice (Figure 4B and 4D) and is lost in hyperplastic mammary glands (n = 4) and mammary adenocarcinomas (n = 6) in these mice (Figure 4C and 4E).

**Figure 4:** Low expression of BRCA2 and Rad51 in cells and mammary tumors deficient for p63 and p73. (A) Western blot analysis for Rad51 using whole cell lysates from wild-type and *p63−/−;p73−/−* MEFs treated with 0 Gy or 10 min (m), 30 m, 1 hour (h), 2 h and 4 h after 5 Gy of gamma irradiation. Actin was used as a control for equal loading. (B–I) Immunohistochemistry (IHC) of normal mammary tissue or mammary adenocarcinomas from *p63+/−;p73+/−* mice using antibodies as follows: (B) normal mammary tissue from *p63+/−;p73+/−* mouse using Rad51 antibody, (C) mammary adenocarcinoma from *p63+/−;p73+/−* mouse using Rad51 antibody, (D) normal mammary tissue from *p63+/−;p73+/−* mouse using BRCA2 antibody, (E) mammary adenocarcinoma from *p63+/−;p73+/−* mouse using BRCA2 antibody, (F) normal mammary tissue from *p63+/−;p73+/−* mouse using p63 antibody, (G) mammary adenocarcinoma from *p63+/−;p73+/−* mouse using p63 antibody, (H) normal mammary tissue from *p63+/−;p73+/−* mouse using p73 antibody, (I) mammary adenocarcinoma from *p63+/−;p73+/−* mouse using p73 antibody.

### p63 and p73 bind to the promoter regions of *Rad51*, *BRCA2*, and *mre11*

Both the cDNA microarray and real-time RT-PCR data provide evidence that *BRCA2*, *Rad51*, and *mre11* are transcriptionally regulated by p63 and p73 after DNA damage (Figure 3). Consequently, chromatin immunoprecipitation (ChIP) assay was performed to determine whether p63 and/or p73 could directly bind to the promoter region of these two genes. A subset of putative binding sites identified and summarized in Table 1 were assayed using ChIP. Sites chosen included those with the best scores for p53 and p63. Four putative binding sites were assayed for *RAD51* (Table 1). RAD51-1 and 2 are located in intron 1, upstream of the start site, while RAD51-3 and 4 are found in intron 2, downstream of the start site. One putative element was assayed for *BRCA2* in intron 2, 133 nucleotides downstream of the start site (Table 1). Lastly, three putative *p53* family response elements were queried for *mre11*: MRE11-1, 2, and 3, located in intron 1, upstream of the start site (Table 1).

ChIP analysis was performed using an antibody for p53, p63 or p73 in wild-type, *p53−/−*, *p63−/−*, and *p73−/−* E1A MEFs treated with doxorubicin for 12 hours (Figure 5). Interestingly, p73 was the only p53 family member that binds to the *RAD51* promoter after DNA damage treatment. p73 was found to bind to RAD51-2 and 3 in intron 1 and intron 2 respectively. The primers used for this PCR reaction did not distinguish between the two sites; therefore, it is possible that p73 only binds to one of these sites. p63 and p73, but not p53, were found to bind to the response element in *BRCA2* after DNA damage (Figure 5). Lastly, p63 was the only family member found bound to the mre-11 promoter at site mre11-3 within intron 1, 171 nucleotides upstream of the start site. The same binding pattern in the ChIP assay was obtained with other DNA damaging agents, such as gamma radiation (data not shown).

**Figure 5:** p63 and/or p73 bind to intronic regions within genes involved in DNA repair. Chromatin immunoprecipitation (ChIP) analysis using wild-type E1A MEFs (WT) and E1A MEFs deficient for the *p53* family members (*p53−/−*, *p63−/−* and *p73−/−*) before (U) and after treatment with doxorubicin (D) for 12 hours. Antibodies used to immunoprecipitate protein-DNA complexes in each cell line are shown in various colors: p53 (red), p63 (blue), and p73 (green). Total input chromatin is shown for each sample (input). Each ChIP was performed using 3 independent MEF lines in triplicate.

### ΔNp63 and ΔNp73 transactivate *Rad51*, *BRCA2*, and *mre11* promoters

The ChIP results clearly demonstrate that p63 and/or p73 can bind to the promoters of these genes; however to gain a clear indication of which isoforms of p63 and p73 transactivate *Rad51*, *BRCA2*, and *mre11*, luciferase assays were performed with TA and ΔN isoforms of *p63* and *p73*. Regions shown to bind by ChIP assay were used to construct firefly luciferase reporters. pGL3-Rad51-1 was designed by cloning intron 1 containing RAD-51-1 and 2 (Table 1) in to the pGL3 basic vector and pGL3-Rad51-2 containing the elements, RAD51-3 and 4, was cloned in to the pGL3 basic vector. These constructs were transfected in to *p63−/−;p73−/−* MEFs along with a renilla luciferase gene and one of the following isoforms of *p63* or *p73*: TAp63α, TAp63γ, TAp73α, TAp73β, ΔNp63γ, ΔNp73α, and ΔNp73β. Interestingly, both ΔNp63α and ΔNp73β are the isoforms that transactivate the Rad51 reporter gene to appreciable levels. ΔNp63α transactivates pGL3-Rad51-1 11 fold and ΔNp73β transactivates this reporter 6 fold (Figure 6A). These isoforms more modestly transactivate the pGL3-Rad51-2 reporter indicating that the p63/p73 element resides in intron 1 (Figure 6A and 6B). Surprisingly, the TA isoforms did not transactivate the reporter gene. The p63/p73 family members also transactivate this reporter gene. ΔNp63α and ΔNp73β together can transactivate the Rad51-1 reporter 19 fold (Figure 6A and 6B). Additionally, the other ΔN isoforms that modestly transactivate this reporter alone can transactivate this reporter to higher levels. For example, ΔNp63α along with ΔNp73α can transactivate this reporter gene 9.8 fold, demonstrating additive effects between these family members.

**Figure 6:** ΔN isoforms of *p63* and *p73* transactivate Rad51 and BRCA2 luciferase reporter genes. Bar graphs showing fold induction for each luciferase reporter gene in (A–D) *p63−/−; p73−/−* or (E,F) *p53−/−;p73−/−* primary MEFs. Reporter genes used are as follows: (A,E) pGL3-Rad51-1 containing the binding elements in intron 1, (B) pGL3-Rad51-2 containing the binding elements in intron 2, (C,F) pGL3-BRCA2 containing the binding element in intron 2, and (D) pGL3-mre-11 containing the binding element in intron 1. Pluses above each bar graph indicate which isoforms of *p63* or *p73* were transfected in cells with the firefly-luciferase reporter genes. Renilla-luciferase was used as a control for transfection efficiency, and pPERP-luc was used as a positive control. Each experiment was performed 6 times using 3 independent MEF lines. Data are represented as the mean ± SEM.

Similar to the experiments for RAD51, the BRCA2 region within intron 1 found to be bound by both p63 and p73 was cloned in to the pGL3 basic vector. Dual-luciferase reporter assay was performed in *p63−/−;p73−/−* MEFs as described above. Strikingly, the isoform with the highest ability to transactivate this reporter was ΔNp73β with a 4 fold induction. Additionally, ΔNp63α and ΔNp73β can transactivate the reporter 6 fold and other combinations of ΔN isoforms also show increases in transactivation of this reporter (Figure 6C).

The ability of p63 and p73 to transactivate the *mre11* gene was also tested by luciferase assay. The region shown to bind to p63 by ChIP analysis was cloned in to the pGL3 basic vector to generate pGL3-Mre11. This reporter was induced 3.8 fold by ΔNp63α and ΔNp73β together (Figure 6D). pPERP-luc, which has previously been shown to be responsive to TAp63γ was used as a positive control for these experiments [23],[24].

To determine whether p53 could transactivate these reporters, p53 was transfected with each reporter and luciferase activity was measured. p53 did not induce any of the reporters assayed (Figure 6A–6D). In addition, we performed luciferase assays using the Rad51-1 and BRCA2 reporters in MEFs lacking *p53*, *p53−/−;p73−/−* (Figure 6E and 6F) and *p53−/−;p63−/−* (data not shown). These experiments yielded similar results as those shown in Figure 6A and 6C. Taken together, these data indicate that the trasactivation of *Rad51*, *BRCA2*, and *mre11* is p53-independent.

### Loss of *p63* and *p73* impairs DNA repair

*Rad51* and *BRCA2* are both involved in homologous recombination (HR) DNA repair, one of the major pathways for repair of double strand breaks (DSBs). Cells lacking genes involved in HR, like *BRCA2* and *Rad51*, have been shown to have an impaired ability to repair their DNA [18],[25],[26],[27]. Consequently, we hypothesized that cells lacking *p63* and/or *p73*, which have low levels of these two proteins, may have a defect in repairing DSBs in damaged DNA. To test this hypothesis, wild-type, *p53−/−*, *p63−/−*, *p73−/−*, and *p63−/−;p73−/−* primary and E1A MEFs were treated with 5 Gy gamma-radiation or doxorubicin to generate DSBs. A comet assay was then performed to determine the DSB repair capacity in these cells. Comet assay, or single cell gel electrophoresis, is a commonly applied approach for detecting DNA damage in a single cell. The unwound, relaxed DNA migrates out of the cell during electrophoresis and forms a “tail” [28]. Therefore, cells that have damaged DNA appear as comets with tails containing fragmented and nicked DNA, while normal cells do not. The degree of DNA damage is represented using the parameter known as tail moment defined as the product of the tail length and the portion of total DNA in the tail. MEFs lacking the *p53* family members were treated with DNA damage and incubated for a total of 16 hours allowing the homologous recombination repair to take place. Cells were and harvested at 0 (untreated), 1, and 16 hours for the Comet assay. In all cases, *p63−/−*, *p73−/−*, and *p63−/−;p73−/−* MEFs were found to have the largest tail moment after DNA damage (Figure 7A–7D). The tail moment after DNA damage was significantly higher for *p63−/−*, *p73−/−*, and *p63−/−;p73−/−* primary and E1A MEFs (18.8) compared wild-type samples (p <0.0001). This result indicates that *p63* and *p73* play a critical role in DNA repair.

**Figure 7:** Cells deficient for *p63*, *p73*, or both *p63* and *p73* have an impaired ability to repair damaged DNA and exhibit increased sensitivity to ionizing radiation. (A–D) DNA damage (tail moment) detected by the Comet assay at 0 (untreated), 1, and 16 hours in E1A MEFs treated with (A) 5 Gy γ radiation, (B) 0.34 µM doxorubicin or primary MEFs treated with (C) 5 Gy γ radiation, and (D) 0.34 µM doxorubicin. Genotypes are indicated on the x-axis and tail moment is shown on the Y-axis. Three independent MEF lines were assayed for each genotype in triplicate. Asterisks indicate statistical significance compared to wild-type (p <0.0001). (E,F) Clonogenic survival of E1A MEFs of the indicated genotypes following (E) gamma radiation and (F) doxorubicin. (G,H) Clonogenic survival of primary MEFs of the indicated genotypes following (G) gamma radiation and (H) doxorubicin. Percent (%) survival is indicated on the Y-axis for each dose of gamma-irradiation (0, 1, 2, 3 Gy) or doxorubicin (0.34, 0.5, 1 µM) on the x-axis. Three independent MEF lines were assayed for each genotype in triplicate. Data are represented as the mean ± SEM.

### Loss of *p63* and *p73* reduces cell survival

Because loss of *p63* and *p73* impair DSB repair by regulating *Rad51*, *BRCA2*, and *mre11*, it is likely that loss of *p63* and *p73* results in poor cell survival due to the inability to repair damaged chromosomal DNA. To determine whether loss of *p63* and *p73* results in a decrease in cell survival, a clonogenic survival assay was performed using both primary MEFs and E1A expressing MEFs after treatment with 1, 2 and 3 Gy of gamma radiation and 0.34, 0.5, and 1.0 µM doxorubicin. After 12 hours, cells were replated and assayed for the ability to form colonies. *p63−/−;p73−/−* E1A MEFs and primary MEFs have an impaired ability to form colonies after gamma radiation indicative of defects in DNA repair (Figure 7E and 7F). A similar result was seen after treatment with doxorubicin in these cells (Figure 7G and 7H).

## Discussion

p53 transactivates a vast network of genes in response to DNA damage [1]. While p63 and p73 can also transactivate known p53 target genes to varying degrees, they play roles in distinct biological functions including development and metastasis and likely have unique transcriptional targets. The advantage of the system employed here is the use of isogenic primary cells with the deletion of a single *p53* family member. Here, we used early passage MEFs lacking the *p53* family members individually or both *p63* and *p73* in combination and expressing E1A, which sensitizes them to undergo apoptosis after DNA damage to identify changes in gene expression in this process. We identified sets of genes that are regulated by individual and multiple p53 family members indicating unique and overlapping functions for this family of genes in response to DNA damage. Six hundred twenty out of 15,488 genes queried were regulated by a p53 family member. Genes identified played a role in multiple processes including apoptosis and DNA repair. In addition to engaging pathways predicted to be induced by DNA damage, genes involved in other processes like development and metastasis were also induced. These are biologically significant given the reported developmental, tumor, and metastatic phenotypes of the *p63/p73* mutant mice [7],[20],[22],[29]. Lastly, the majority of the targets identified had binding sites that closely fit the p53 and p63 consensus binding site [14],[30],[31] indicating that they may be *bona fide* direct transcriptional targets of these family members. Indeed, we verified that *Rad51*, *BRCA2*, and *mre11*, genes involved in DNA repair, are direct transcriptional targets of p63 and p73.

Given the high prevalence of mammary adenocarcinoma in mice mutant for *p63* and *p73* (*p63+/−;p73+/−*), a group of genes of interest are those involved in DNA repair. These genes were induced in wild-type cells and down regulated in the absence of *p63* or *p73*. The mechanism for the tumor suppressive activity of *p63* and *p73* is not completely understood [6],[7],[32]. Regulation of DNA repair genes by p63 and p73 has not been demonstrated previously and could be a pathway employed by these genes in tumor suppression. Both Rad51 and BRCA2 were found to be direct transcriptional targets of p63 and p73 indicating that these mechanisms may be triggered during tumorigenesis. Interestingly, Rad51 has been shown previously to be repressed by p53 through a site found upstream of the start site [33]. Here, we show that ΔNp63 and ΔNp73 transactivate Rad51 through a distinct element in intron 1 indicating that there is an intricate and complex regulation of this gene by the p53 family and is likely a critical target in tumor suppression by this family. We also showed that transcriptional regulation of *Rad51*, *BRCA2*, and *Rad51* by p63 and p73 is p53-independent/

It was surprising that the ΔN isoforms of p63 and p73 were more potent transactivators of *Rad51*, *BRCA2*, and *mre11* than the TA isoforms. The TA isoforms have an acidic N-terminal domain necessary for transactivation [2],[3], and many studies have shown previously that the TA isoforms are more potent transactivators than the ΔN isoforms [2],[8]. Furthermore, the ΔN isoforms are better known for the dominant negative activities that they impose on the TA isoforms of *p63* and *p73* and *p53*. Interestingly, a number of recent studies have shown that the ΔN isoforms are capable of transactivating target genes due to a proline-rich transactivation domain that exists in these isoforms [12],[13]. In addition, the ΔN isoforms of *p63* are more highly expressed than TAp63 in certain tissues including the skin [14] making the ΔNp63 isoforms likely candidates for gene regulation in these tissues. Taken together, our results indicate that the roles of the ΔN isoforms are more complex than previously appreciated.

We have shown previously that E1A expressing MEFs deficient for *p63* and *p73* are resistant to apoptosis [15]. Paradoxically, we found that *p63−/−;p73−/−* primary and E1A MEFs are radiosensitive in long-term clonogenic assays. This finding coupled with the inability of *p63/p73* deficient cells to repair DNA as shown by Comet assay indicate that *p63* and *p73* play a critical role in DNA repair. This new finding does not preclude that *p63/p73* deficient cells are resistant to apoptosis after acute exposure to DNA damage. These data demonstrate that surviving *p63−/−;p73−/−* cells are unable to proliferate and establish a colony after DNA damage. This is likely due to defects in the DNA repair mechanisms.

Using a genome wide analysis, these studies have revealed novel transcriptional targets of the *p53* family members. We have also identified a novel mechanism of the regulation of the DNA repair pathway by *p63* and *p73*. Given the high incidence of mammary adenocarcinoma in *p63/p73* mutant mice, these studies have unveiled a potential mechanism for *p63* and *p73* as tumor suppressor genes. In addition, our studies have revealed further complexity by indicating that the primary transactivators of these DNA repair genes are the ΔN isoforms of *p63* and *p73*. These isoforms have previously been thought to act as oncogenes. More recent data have challenged this notion as these isoforms can also transactivate genes involved in apoptosis and the expression of these isoforms does not provide a growth advantage [12]. These studies provide further evidence that the ΔN isoforms may have some anti-tumor functions such as the ability to engage DNA repair pathways. Future studies using isoform specific knock out mice should yield important insights in to how each of these isoforms contributes to tumor suppression and shed light on the interactions of the complex *p53* family.

## Materials and Methods

### Preparation of 15 K murine cDNA microarrays

The Laboratory of Genetics at The National Institute on Aging (NIA) cloned approximately 15,000 unique cDNAs into the NotI/SalI site of Ampicillin-resistant pSPORT1 vector (Life Technologies). Average insert size of the clones is 1.5 kb (0.5–3 kb). Inserts were amplified for microarray printing following a modified version of the protocol described previously [34]. In 96 well format, bacterial stocks were grown overnight in 2X YT medium (100 µg/ml ampicillin) with agitation. Ten microliters of the overnight bacterial culture was added to 90 µl ddH_2_O in PCR plates (MJ Research) and denatured at 95° C for 10 minutes. Following denaturation, plates were centrifuged for 10 minutes. To perform PCR, 5 µl of supernatant from each well was used as template in a 100 µl reaction with 3.5 units of AmpliTaq DNA polymerase (Applied Biosystems), forward primer (5′–CCAGTCACGACGTTGTAAAACGAC-3′) reverse primer (5′-GTGTGGAATTGTGAGCGGATAACAA-3′), and deoxynucleotide triphosphates (dNTPs). Amplification was carried out in thermocyclers with a program that contained an initial denaturation step at 95°C for 2 minutes followed by 38 cycles of 30 s at 94°C, 45 s at 65°C, and 3 minutes at 72°C, and a final extension of 5 minutes at 72°C. The amplified inserts were then purified using Montage PCR_96_ cleanup Filter Plates (Millipore) on a BIO-TEK Precision 2000 Automated Microplate Pipetting System to a purified volume of 100 µl. Thirty-five microliters of each purified PCR product was added to a 384-well plate, and desiccated using a large Savant Speed-vac apparatus, then reconstituted in 7 µl of 3X SSC/1.5 M betaine to a mean concentration of 600 ng/µl. The microarrays were fabricated at the MIT BioMicro Center using Corning GAPS II Gamma Amino Propyl Silane slides. cDNA clones were printed using a BioRobotics Microgrid 600 TAS Arrayer with a 32-pin print head and quill pin microfluidic liquid transfer technology.

### Cell culture, RNA extraction, and labeling of the cDNA probe

All procedures involving mice were approved by the IACUC at U.T. M.D. Anderson Cancer Center and M.I.T. E1A-expressing mouse embryonic fibroblasts (MEFs) (wild-type, *p53−/−*, *p63−/−*, *p73−/−*, and *p63−/−;p73−/−*) were generated as described previously [15] from passage 1 primary MEFs. 3×10^6^ E1A MEFs were plated on each of 6–15 cm dishes. Twenty-four hours after plating, the cells were treated with 0.34 µM doxorubicin. Twelve hours after treatment, total RNA (150–300 µg) was extracted from treated and untreated E1A MEFs using the RNAeasy Midi Kit (Qiagen). For each microarray hybridization, 100 µg of total RNA prepared from the reference or experimental cells were labeled by incorporating Cy3- or Cy5-labeled dUTP (NEN) using oligo d(T) (MWG) and Superscript II reverse transcriptase (Invitrogen). The resulting probes were purified using the Qiaquick PCR purification Kit (Qiagen) and recovered in a volume of 30 µl ddH_2_0.

### Microarray hybridization

The printed slides were rehydrated, UV cross-linked, and blocked to reduce background using succinic anhydride (Sigma), 1-methyl 2-pyrrolidinone and sodium borate. Each slide was incubated in 60 µl total volume of hybridization solution containing Cy3- and Cy5-labeled target (one probe is the reference invariant target and the other is the experimental target), 1 µg of Mouse Cot-1 DNA (Invitrogen), 0.1 units of poly-A_40–60_ (Amersham Pharmacia), and 10.1 µg of Salmon Testes DNA (Sigma), 25% Formamide, 5X SSC, 0.1% SDS under a 22×40-mm lifterslip (Erie Scientific Company) at 42°C for 16 hours exactly. The slide was placed in a sealed hybridization chamber (Corning) containing two side wells with a total of 20 µl 3X SSC for humidification in a light-sealed water bath. After exactly 16 hours of hybridization, the slide was washed in 500 ml of 1X SSC, 0.03% SDS for 5 minutes after the lifterslips are gently removed in the wash solution. Then, the slides were washed for 5 minutes in 0.1X SSC, 0.01% SDS followed by 0.1X SSC. Slides were centrifuged in a speed-vac to dry. Each slide was scanned using an arrayWoRx Auto Biochip Reader that employs white light, polychromatic filter-wheel/CCD camera (Applied Precision) at wavelengths corresponding to each analog's emmision wavelength (595 and 685 nm for Cy3 and Cy5, respectively). RNA from each sample was hybridized to four independent cDNA microarrays. For 2 replicates, the invariant target was labeled with Cy3 and the experimental target was labeled with Cy5. For the other 2 replicates for each sample, the invariant target was labeled with Cy5 and the experimental target was labeled with Cy3. The invariant reference target RNA used was extracted from untreated wild type- E1A MEFs. These cells were chosen as a source of reference target RNA because this species of RNA robustly hybridized to a large percentage of genes, and it is relevant to the experimental design.

### Data processing

#### Hierarchical mapping

Microarray images imported from the arrayWoRx scanner were filtered and annotated using the DigitalGenome software (MolecularWare). The resulting spot intensity data was normalized using the rank invariant method [35]. The gene filtering process was performed using SAM [16]. SAM is a statistical technique designed for analysis of microarray data [16] that uses repeated permutations of array data to report the most statistically significant differentially expressed genes between two groups of samples. Using all four microarray replicates, SAM reports an estimate of the median false discovery rate (FDR) for each list of differentially expressed genes. The FDR is the percentage of genes falsely reported as showing statistically significant differential expression. In addition, SAM uses an algorithm based on the Student *t*-test to determine the q-value of each individual gene, which is the lowest FDR at which the gene is called significant [36]. Using the *bona fide* biological target of p63, *PERP*, we used a cut-off FDR of 8.24% to determine our list of significant genes. As a result, 15 genes on our list has a q-value between 5% and 8.24% while the remaining 605 genes have a q-value less than 5%. Heatmaps were generated using functions within the Bioconductor project [37] of the R statistical programming language. Background subtracted and normalized intensity values obtained from the microarray experiment comparing the different cell populations were used. To perform hierarchical clustering of the genes and cell samples, Euclidean distance was used to compute dissimilarity.

#### Identification of p53/p63 binding sites

To identify all potential p53-family binding sites, promoter sequences (defined as genomic sequences within 2 kb of the transcription start site which have previously been reported to be enriched for these sites [30]) and intron 1 were extracted for all genes regulated by each p53 family member. These promoter sequences were initially searched for CWWG tetramers separated by a spacer of 5–8 nucleotides. To increase the specificity and score of these predicted sites, both strands were searched with a series of position-specific matrices for p53 [30],[31],[38] and p63 [14],[39] using HMMER1 v1.8 [17] with the “local search” option. To rank sites predicted across multiple matrices, all CWWG tetramer pairs were matched to corresponding HHMER sites and scored using the sum of bit scores.

### Quantitative Real Time PCR

Total RNA was extracted from the E1A MEFs of the genotypes described above using the RNeasy Midi and Rnase-free Dnase kits (Qiagen). RNA was quantified and tested for quality on the Agilent 2100 Bioanalyzer (Agilent Technologies). To generate cDNA, RNA (2 µg) from each E1A MEF line treated with 0.34 µM doxorubicin was used for random hexanucleotide- primed cDNA synthesis. Each 40 µl reaction contained 1X buffer, 10 µM DTT, 1 µg random hexamer, 2 µl of Superscript II (Invitrogen), 0.5 mM each of all four dNTPs, and 80 units of RNase inhibitor (Promega). Using heating blocks, reactions were incubated at 42°C for 1 hour, 70°C for 15 minutes, 37°C for 20 minutes, and 95°C for 2 minutes. RNase H (2 units) (Invitrogen) was added to each reaction following the 70°C incubation. Afterwards, each reaction was diluted with ddH_2_O to a final working volume of 200 µl. cDNAs (2 µl) were added to 25-µl reaction mixtures containing 12.5 µl of 2X SYBR Green master mix (Applied Biosystems), and 40 nm of gene-specific primers. Primers were designed using Primer Express software (Applied Biosystems). Assays were performed in triplicate with an ABI Prism 7000 Sequence Detector (Applied Biosystems). All data were normalized to an internal standard (18 S ribosomal RNA; TaqMan Ribosomal RNA Control Reagents VIC Probe: Protocol: Rev C, Applied Biosystems) or GAPDH.

### Chromatin Immunoprecipitation Assay

ChIP Assay was performed as described previously, E1A MEFs (wild-type, *p53−/−*, *p63−/−*, *p73−/−*, and *p63−/−;p73−/−*) were untreated or treated with 0.34 µM doxorubicin for 12 hours, which are the same conditions used for the array and real time PCR. Cellular proteins were crosslinked to chromatin with 1% formaldehyde. p53-DNA, p63-DNA or p73-DNA complexes were immunoprecipitated using the following antibodies: pan-p63 (4A4, Santa Cruz), pan-p73 (IMG-259a, Imgenex) or p53 (Ab-3, Oncogene Research Products). Immunprecipitated complexes were recovered by *Staphylococcus A* cells, treated with proteinase K, and DNA was purified. PCR was performed for putative p53 family binding elements. Putative p53 family member binding sites were identified by scanning 1000 bp of the 5′ UTR, exon 1, intron 1, exon 2 and intron 2 for the consensus p53 binding site [31]. These sites are summarized in Table 1. Sequences for primers used are available upon request.

### Construction of luciferase reporters

To generate the pGL3-Rad51 luciferase reporter, DNA was amplified from a BAC clone containing the Rad51 gene (RP23-15121, CHORI BACPAC resources) using primers designed containing the p73 binding site shown by ChIP and 5′ NheI and 3′ XhoI cloning restriction enzyme sites: forward primer (5′- ACTAGCTAGCAGCAGGGCGACCAACCGAC-3′) and reverse primer (5′-CCGCTCGAGTGGCCCTCCCTATCCACAGG-3′). To construct the pGL3-BRCA2 luciferase reporter, the DNA fragment containing the p63/p73 binding site shown by ChIP was amplified from C57/B6 genomic DNA by PCR using the following primers with 5′ XhoI and 3′ BglII cloning restriction enzyme sites: forward primer (5′-CCGCTCGAGAGAGGGATCCGGCGCGTC-3′) and reverse primer (5′-GGAAGATCTGGTCTAAGCTCTGTTGCTCCTG-3′. To generate the pGL3-Mre11 luciferase reporter, DNA was amplified from a BAC clone containing the mre11a gene (RP23-149D5, CHORI BACPAC resources) using primers designed containing the p63 binding site shown by ChIP and 5′ XhoI and 3′ BglII cloning restriction enzyme sites: forward primer (5′- CCGCTCGAGACAGAGAGAACCTCACCGAGAAC -3′) and reverse primer (5′-GGAAGATCTCTGTACCAGGTTCCTCTCCAAG-3′). The resulting amplified DNA fragments were gel-purified (Wizard Prep Kit, Promega) after restriction enzyme digestion and then ligated to pGL3-basic vector (Promega) between the respective cloning sites.

### Western blot analysis

6×10^5^ wild-type and *p63−/−;p73−/−* MEFs were plated on 6 cm dishes. Twelve hours after plating, the MEFs were irradiated with 5 Gy of gamma-irradiation and then harvested at 10 minutes, 30 minutes, 1, 2, and 4 hours. The MEFs were lysed on ice in lysis buffer (100 mM Tris, 100 mM NaCl, 1% Nonidet P40, protease inhibitor cocktail (Roche)). Thirty micrograms of each lysate was subjected to electrophoresis on a 10% SDS PAGE for Rad51 and transferred to PVDF membrane. Rad51 was detected using the anti-Rad51 antibody (clone 51RAD01, Neomarkers), and BRCA2 was detected using the anti-BRCA2 antibody (clone H-300, Santa Cruz).

### Immunohistochemistry

Slides were dewaxed in xylene and rehydrated in a graded series of ethanol following standard protocols [7]. Slides were incubated with primary antibodies for p63 (4A4, Santa Cruz), p73 (IMG-259A, Imgenex), Rad51 (clone 51RAD01, Neomarkers), or BRCA2 (clone H-300), Santa Cruz). at a dilution of 1∶100 for 18 hours at 4 deg C. Detection was performed using the Vectastain kit (Vector Labs) followed by the VIP kit or DAB kit (Vector Labs) and counterstained with methyl green (Vector Labs). Ten normal mammary glands and ten mammary adenocarcinomas were stained with each antibody.

### Dual-luciferase reporter assay

*p63−/−;p73−/−*, *p53−/−;p73−/−* or *p53−/−;p63−/−* MEFs were plated on 6-well plates (3.5×10^5^ cells per well). Twelve hours after plating, the MEFs were transiently transfected using Fugene HD (Roche) with 2.5 µg of the following Firefly luciferase reporter plasmids (pGL3-Rad51-1, pGL3-Rad51-2, pGL3-BRCA2) or pPERP-luc [24], 1 µg of Renilla luciferase plasmid (transfection control), and 2.5 µg of empty vector (pcDNA3) or plasmids encoding the p63/p73 isoforms (TAp63α, TAp63γ, ΔNp63γ, TAp73α, TAp73β, ΔNp73α and ΔNp73β) or p53/ In experiments where 2 isoforms of p63 and p73 were assayed simultaneously, 1.25 µg of each isoform was used. After 24 hr, cells were harvested and luciferase activity was measured using the Dual-Luciferase Reporter Assay system (Promega) and a Veritas microplate luminometer (Turner BioSystems). The relative luciferase activity was determined by dividing the Firefly luciferase value with the Renilla luciferase value and the fold increase in relative luciferase activity was determined by dividing the relative luciferase value induced by p63 and p73 isoforms with that induced by the pcDNA3 control vector. Each experiment was performed in triplicate.

### Clonogenic survival assay

E1A MEFs or primary MEFs were plated in 6-well plates (1×10^6^ cells per well) of the following genotypes (wild-type, *p53−/−*, *p63−/−,p73−/−*, and *p63−/−;p73−/−*) [15]. Twelve hours later, MEFs were irradiated with 1, 2, and 3 Gy of gamma radiation or 0.34, 0.5, and 1 µM doxorubicin. After 12 hr, 1200 cells were plated on 10 cm dishes. After 12 days of incubation, the cells were stained with clonogenic reagent (0.25% of 1,9-dimethyl-methylene blue in 50% ethanol). Surviving colonies were counted, and the survival rate was calculated as the ratio of the surviving colonies after DNA damage treatment over the number of colonies for each genotype before treatment. Each experiment was performed in triplicate on three independent MEF lines for each indicated genotype.

### Comet assay

Wild-type, *p53−/−*, *p63−/−*, *p73−/−*, and *p63−/−;p73−/−* primary and E1A MEFs were plated on 6-well dishes (1.6×10^5^ cells per well). Twelve hours after plating, MEFs were irradiated with 5 Gy of gamma radiation. Cells were harvested 0,1, and 16 hours later for Comet Assay (Trevigen) according to the manufacturer's protocol specific for DSB detection. Briefly, cells were suspended in PBS at a density of 3×10^5^ cell/mL. Twenty microliters of each cell suspension was mixed with 200 µL of melted low melting point agarose (LMA) and 75 µL of this mixture was placed onto the Trevigen CometSlide for electrophoresis. Subsequent to electrophoresis, samples were visualized with SYBR Green I and fluorescence microscopy. Twenty pictures were taken for each sample and at least 135 cells per experiment were examined for comet tails using CometScore software (TriTek Corporation). Three independent MEF lines for each genotype were assayed in triplicate. Student's t test was used for statistical analysis.

### Statistics

All experiments were performed at least in triplicate. Data are represented as the mean ± SEM. Statistics for qRT-PCR, luciferase, clonogenic, and comet assays was performed using Student's t test for comparison between two groups. A p value of 0.05 was considered significant.

## Supporting Information

Figure S1 Heatmap showing unsupervised hierarchical clustering analysis of *p53*, *p63*, and *p73−/−* E1A MEFs after doxorubicin treatment. Each row represents the relative expression level for a gene compared to an untreated isogenic MEF line. The columns represent multiple isogenic MEF lines for each indicated genotype. Only genes that were significantly down-regulated in at least one mutant MEF line and not wild-type MEFs in response to doxorubicin treatment are represented. The red color indicates high expression and the green color indicates low expression, while black indicates no significant change. Clustering based on Euclidean distance indicates that *p63* and *p73* deficient E1A MEFs are more similar to each other than to *p53−/−* E1A MEFs. The GenBank Accession Number is shown in the right hand column.
(0.39 MB PNG)

Figure S2 Genes involved in DNA repair are differentially expressed in MEFs deficient for *p63* and/or *p73*. Real time PCR analysis of E1A MEFs of the following genotypes (wild-type, *p53−/−*, *p63−/−*, *p73−/−*, and *p63−/−;p73−/−*) before and after (D) treatment with doxorubicin. The Y-axis shows the relative mRNA levels of mre11, BRCA2, Rad51, and Rad50 before and after treatment with doxorubicin (0.34 µM) for 12 hours. GAPDH was used as an internal control. Bars represent 3 MEF lines for each genotype, each performed in triplicate. Data represented as mean ± SEM.
(2.17 MB TIF)

Table S1 Pathway analysis of p63 and p73 target genes.
(0.11 MB JPG)

Table S2 Identified p53/p63 binding sites for genes with differential expression.
(1.10 MB XLS)
